The article "Cross-Cultural Validation of Health and Quality of Life Measures for Children in Hong Kong" was published in 2022. Journal: Occup Ther Int.

# Cross-Cultural Validation of Health and Quality of Life Measures for Children in Hong Kong

**DOI:** 10.1155/2022/5672679

**Published:** 2022-09-27

**Authors:** Hiu Lam Helen Sze, Cheuk Lam Beanie Fung, Pui Pui Phoebe Cheung, Tsz Yuk Amy Chim, Ming Ho Lee, Cheuk Chi Cynthia Law, Wui Man Benson Lau

**Affiliations:** ^1^Department of Rehabilitation Sciences, The Hong Kong Polytechnic University, Hung Hom, Hong Kong; ^2^Yew Chung College of Early Childhood Education, Aberdeen, Hong Kong

## Abstract

**Objective:**

The Pediatric Quality of Life Inventory (PedsQL™) 4.0 is a health-related quality of life (HRQOL) measure designed for clinical practice and research, health policy evaluation, and general population surveys. There is a dearth of instruments measuring quality of life in children which are available in Chinese and validated for Chinese populations. Therefore, this study attempted to establish the Hong Kong populations' norms for the Chinese version of PedsQL™ and examined the psychometric properties of the measure for this population.

**Methods:**

Sixty-nine children (aged 7 to 12 years) and their parents completed the child self-report and the parent proxy report, respectively, of the PedsQL™ 4.0 Generic Module. To evaluate construct validity, a group comparison of children with special educational needs (SEN) (*n* = 21) and those with typical development (TD) (*n* = 48) was conducted. Differences based on age group and gender and parent–child agreement on the perception of the child's HRQOL were also examined.

**Results:**

Children with SEN had a lower quality of life perception than those with TD in the physical, social, and schooling domains. No significant differences in emotional health were found between the two groups. The differences between the children with SEN and with TD varied based on age group and gender. The differences between the parents' and children's perceptions of the children's HRQOL were insignificant in this sample.

**Conclusion:**

Norms for the Chinese version of the PedsQL™ 4.0 Generic Module for the Hong Kong population were established in the study, and both the child self-report and parent proxy report were found to be reliable and valid for this population.

## 1. Introduction

The number of studies being conducted on the health-related quality of life (HRQOL) measurements has increased significantly in recent decades [1]. HRQOL refers to “how well a person functions in their life and his or her perceived well-being in physical, mental, and social domains of health” (p. 646). Measurements of HRQOL are important for monitoring population health and evaluating the impact of public health interventions. Such measurements are particularly crucial for identifying at-risk children and adolescents and for detecting hidden comorbidities and healthcare needs before formal medical diagnoses [2]. HRQOL measurements have been widely used for promoting health and behavioral interventions in child and adolescent populations [3]. However, despite the development of numerous HRQOL instruments in Western countries and their validation in those populations, only a few have been applied and validated in the Chinese population.

Assessing patients' quality of life (QoL) is important for healthcare professionals in capturing clients' own perspectives of their diseases and treatment effectiveness. A 2020 study reported that French hospital doctors recognized QoL assessment as a standardized tool to minimize subjectivity and ensure stability of outcome [4]. It is crucial for clinicians in formulating tailored care plans for clients and fostering therapeutic relationships. As healthcare professionals are the main caregivers for hospitalized and institutionalized patients, their perspectives on patients' QoL should be aligned with the patients' QoL [5]. However, several studies have found discrepancies between healthcare professionals' HRQOL evaluations of clients and by the clients themselves [6–9]. Furthermore, a survey conducted by Zidarov et al. [10] found no consensus among healthcare professionals on the outcome measures used for evaluating HRQOL. Therefore, there is an urgent need for evidence-based assessment tools to evaluate HRQOL.

Occupational therapy (OT) practitioners strive to improve the QoL of clients and facilitate their optimal engagement in meaningful life roles and activities [5]. OT intervention helps clients to optimize their occupational performance, which refers to their ability to perform the activities that make up their individual lifestyles [1]. Improvements in occupational performance increase well-being across various life domains, resulting in a higher QoL. Therefore, QoL is used as a key outcome measure in OT interventions [5].

To obtain a valid and standardized HRQOL measure for a population, a prospective measure must first be tested on the population, and the population's norms for the measure must be established. Normative data is needed to determine whether individual scores are above or below the average in one's country or region according to their gender and age [11]. Validated and standardized HRQOL measures can be used to evaluate the impact of illnesses and the effectiveness of treatment as perceived by the general population. They can be used as outcome indicators by clinicians to formulate client-centered and cost-effective healthcare services [12].

The Pediatric Quality of Life Inventory (PedsQL™) 4.0 is commonly used to assess children's HRQOL. The instrument has been translated into numerous languages, including Spanish and Vietnamese [2]. Although the Chinese version of the instrument has been validated in Mainland China and Taiwan, the Hong Kong population's norm for the measure has not yet been established [13, 14]. The Chinese version of the PedsQL™ 4.0 Generic Module was found to be supported for measuring the HRQOL of children with cerebral palsy in mainland China by one study [14]. The Chinese version of the PedsQL™ 4.0 Generic Module was also proved to be reliable and valid for the Taiwanese population [13]. Regarding disease-specific modules, the Cardiac Module and the Diabetes Module of PedsQL™ have been validated in Mainland China [13]. Both of these modules and the Cancer Module have been validated in Taiwan, whereas only the Cancer Module has been validated in Hong Kong [13, 15]. Finally, the reliability and validity of the Generic Module of PedsQL™ 4.0 were supported for measuring HRQOL in boys with Duchenne muscular dystrophy for the Chinese population [16].

This study conducted an initial validation of the Chinese version of Generic PedsQL™ 4.0 for the Hong Kong population. There are two objectives in this study. The first was to compare the QoL of children with typical development (TD) with that of children with special educational needs (SEN) using the generic PedsQL™ 4.0 self-report and parent proxy report. We hypothesized that children with SEN would have lower HRQOL than those with TD both overall and in each subscale. The second objective was to investigate parent–child agreement on perceptions of HRQOL among both children with TD and children with SEN.

## 2. Methods

### 2.1. Overview of the Method

The Chinese version of the generic PedsQL™ was obtained from the official website of PedsQL™. Approval was obtained from the Hong Kong Polytechnic University Ethics Committee (HSEARS20210114002). The parents of the children recruited for the study provided their informed consent to participate in the study and to release the information from their questionnaire results.

### 2.2. Instrument

PedsQL™ 4.0 is a 23-item inventory with a 5-point Likert-type response scale [3]. There are two variants of the inventory: the child self-report to capture the child's perception and the parent proxy report to capture the parents' perception of their child's QoL. The 23 items are divided into four subscales: physical functioning (8 items), emotional functioning (5 items), social functioning (5 items), and functioning at school (5 items). The latter three subscales together represent psychosocial functioning. A study showed that the internal consistency reliability and construct validity of the child self-report and parent proxy report scales meet the minimum standards of alpha coefficients (>0.70) and significance values (*p* < 0.001) [2]. PedsQL™ consists of generic core scales and disease-specific modules. The generic core scales have been used in several studies on various medical conditions. For instance, PedsQL™ has been adopted in the meta-analysis of the QoL of children with chronic kidney diseases and in the investigation of the impact of poverty and differences in family earnings on Hong Kong children's psychological health [17, 18]. PedsQL™ has also been validated for measuring the QoL of young people with autism spectrum disorder and children and young adults with intellectual and developmental disabilities [19, 20].

This study adopted the generic core scales for children aged 7 to 12 years. The generic core scales were used because the student participants with SEN had none of the conditions indicated in any of the established disease-specific modules.

### 2.3. Procedure

The data were collected from April to July 2021. For the collection of data from the TD group, the schools were recruited using stratified sampling according to the primary schools from various geographical regions. One primary school each from Kowloon and the New Territories participated in the data collection, after consent was obtained from the school principals. In each grade in the schools, students were chosen from three categories, namely, *high*, *moderate*, and *low* levels of academic performance, as indicated by their teachers to ensure equal representation across the entire range of academic performance. For the SEN group, the students and their parents were recruited using convenience sampling from a therapeutic group organized by the university from April to May 2021.

Before data collection, the Chinese version of the PedsQL child self-report and parent proxy questionnaires was reviewed by the teachers to improve the clarity and fluency of each item. The participants' sociodemographic information was gathered with a questionnaire. Due to the restrictions by the COVID-19 pandemic, some of the questionnaires were administered online. However, for children with SEN, the data were collected using face-to-face surveys to immediately address any problems encountered by parents and their children. These face-to-face surveys were conducted by year 4 undergraduate occupational therapy students, and academic staff were available for assistance if requested by the students.

### 2.4. Participants

A total of 112 children with TD aged between 7 years and 12 years and 62 parents were initially invited. The criterion for children's inclusion in the study was the ability to read Chinese fluently. Those with confirmed diagnoses were excluded. The final sample of the TD group consisted of 48 children and their parents. For the SEN group, 21 children with SEN aged between 7 years and 12 years were recruited from the therapeutic group. Tables 1 and 2 present the demographic characteristics of both the child and parent participants in the SEN and TD groups. For the SEN group, diagnostic information was listed. As shown in Table 1, the majority of the children with SEN had at least one confirmed diagnosis (61.9%). More than half of the suspected or confirmed diagnoses were either attention deficit hyperactivity disorder (ADHD) or specific learning difficulty (SpLD) (28.9% and 23.8%, respectively). The demographic data of the parents are presented in Table 2. The education levels of over 80% of the parents from the SEN group and 90% from the TD group were junior secondary level or above.

### 2.5. Data Analysis

Responses to each question were converted first into raw scores of 0, 1, 2, 3, or 4 and then into transformed scores of 100, 75, 50, 25, or 0, respectively. IBM SPSS Statistics version 26 was used for data analysis (IBM Corp., Armonk, N.Y., USA). The Mann-Whitney *U* test was used to evaluate the construct validity by comparing, for each subscale and the overall scale, the means of the self-reported QoL scores reported by the children in the TD and SEN groups. The Mann-Whitney *U* test was also used to investigate the agreement between the children's and their parents' perceptions of the children's HRQOL by comparing the means of the physical, psychosocial, and overall scores of the self-report and parent proxy report responses in each group. The internal consistency reliability of the items was assessed for the child self-report and parent proxy report responses using Cronbach's *α*.

## 3. Results

### 3.1. Reliability

Table 3 presents the internal consistency reliability of the scale and its subscales. As shown in the table, the internal consistency reliabilities (Cronbach's *α*) of most of the subscales and the overall scale were acceptable. The exceptions were the self-reports and parent proxy reports of the school functioning subscale for the children with SEN (*α* = 0.480 and *α* = 0.566, respectively). These results indicate that the questions in the schooling subscale were internally inconsistent in depicting the school functioning QoL of children with SEN.

### 3.2. Comparison between SEN and TD Groups

Table 4 presents comparisons of PedsQL between the children with SEN and the children with TD. As shown in the table, the mean scores for the children with SEN were significantly lower than for those with TD in physical (*p* ≤ 0.01), social (*p* = 0.012), and schooling performance (*p* = 0.012) based on the child's self-report. Although there was no significant differences in emotional functioning (*p* = 0.183), there was a significant difference in overall psychosocial health (*p* = 0.015) between the children with SEN and the children with TD. These findings suggest that the children with SEN perceived themselves to have a poorer HRQOL than their peers with TD, except in the domain of emotional functioning.

The differences in PedsQL between the children with SEN and TD groups in each age group and gender were also explored.  Table 5 presents the age differences in HRQOL between the children with SEN and TD. As shown in the table, the junior age group (ages 7–8) of children with SEN and children with TD demonstrated a significant difference only in physical health (*p* = 0.008). For the senior age group (ages 9–12), significant differences were found between the children with SEN and the children with TD in physical health (*p* = 0.034), social functioning (*p* = 0.001), and psychosocial health (*p* = 0.034) and on the overall scale (*p* = 0.023). These results suggest that the HRQOL of the children with SEN was significantly worse than that of the children with TD on more subscales for the senior age group.  Table 6 presents the gender differences in PedsQL between the children with SEN and TD. The female group with SEN demonstrated statistically lower scores in social functioning (*p* = 0.025) than those with TD. Greater differences were found in the subscales of physical health (*p* = 0.002), school functioning (*p* = 0.001), and psychosocial health (*p* = 0.020) and the overall scale (*p* = 0.006) ips.

### 3.3. Parent–Child Agreement on the Perceptions of Children's QoL

Table 7 illustrates the agreement between the parents and their children's PedsQL in each group. No significant difference was found in the TD group across the scales of physical (*p* = 0.173), psychosocial (*p* = 0.820), and overall functioning (*p* = 0.873). Similarly, no significant difference was found in the SEN group between the parents' and children's perceptions of physical (*p* = 0.478), psychosocial (*p* = 0.066), and overall performance (*p* = 0.378). These results indicate that the parents' and children's perceptions of the children's QoL were similar. However, significant differences might have been found in perceptions of school functioning between the parents and children in the SEN group which had the sample size been larger, as the *p* value for this comparison (*p* = 0.058) was close to a significant level. This finding suggests that in the SEN group, the parents' perceptions of their children's school functioning were inconsistent with the children's perceptions. Overall, despite the lack of statistical significance of these results, the differences in the mean scores between the child self-report and the parent proxy report responses indicate that in the SEN group, the parents might have underestimated their children's QoL or the children might have overestimated their own QoL.

## 4. Discussion

This study is aimed at establishing the Hong Kong population's norms of the Chinese PedsQL™ 4.0. The QoL of the children and parent proxy with TD was collected. The psychometric properties of the Chinese PedsQL™ 4.0 was evaluated by comparing the age and gender differences of the norm with a group of children with SEN. This study revealed some interesting findings which will be discussed in the following.

### 4.1. Internal Consistency Reliability

The internal consistency of all the items of the Chinese version of PedsQL was within the acceptable range for both the self-report and parent proxy reports, except the school functioning items. The factor loadings among the five items of this subscale were low, indicating that the items did not consistently reflect QoL in terms of school functioning for the children with SEN. One possible reason for this lack of consistency may be the overlap of the PedsQL items with various developmental disabilities. One previous study found that there were some overlapping between items on school functioning scale and ADHD symptoms [20]. Wordings of items such as “being unable to pay attention in class” and “forget about things” resemble descriptions of ADHD symptoms and may therefore assess the attention of children with other diagnoses instead of QoL.

### 4.2. Comparison of PedsQL Age and Gender Differences between the SEN and TD Groups

We found that QoL of children with SEN was generally lower than reported for the norm population, especially on the physical health scale. The academic performance of children with SEN may be affected by their behavioral manifestations of diagnoses. Limitations in the attention capacity of children with ADHD may adversely affect their school performance. Reading and writing difficulties may affect the academic achievement of children with SpLD, thus affecting their QoL in school functioning. The results are consistent with other studies that have reported children with SEN are more prone to have sleep problems as compared to their peers [21]. It has been reported that children with ADHD are more likely to have increased sleep latency, fragmentation, and wakening. Thus, the quality of sleep experienced by children with SEN may adversely affect their physical functioning. Similarly, sleep problems for children with SpLD were noted as they may encounter difficulty in reading and writing in the competitive learning environment in Hong Kong. In order to cope with the heavy school work, they may have less time to sleep and play which subsequently decreases their physical performance over the long term. Moreover, poor executive function in children with SEN may negatively affect their planning and organization and lead to difficulties in initiating and maintaining activities [22]. In one study, children with ADHD and SpLD participated less in physical activities and organized sports because of weaker executive functioning and hence perceived themselves as lower in the physical functioning.

Moreover, children with SEN may have difficulty integrating with their peers which could reflect lower scores in social functioning. Due to the impulsive and intrusive symptoms exhibited by children with ADHD, they may have difficulty engaging in social exchanges such as turn-taking and cooperation [23]. When provoked, they may express hostile emotions more explicitly than peers with typical development. With such behavioral problems, children with ADHD may be rejected by their peers and have fewer reciprocal relations, resulting in reduced social functioning [24]. Children with SpLD, who generally experience learning difficulties and have poorer academic results than their peers with typical development, may be labelled as low achievers in schools [25]. The social stigma associated with low academic achievement may adversely affect their self-esteem. This feeling of inferiority among children with SpLD may cause low self-efficacy in social interactions with their peers, thus affecting their social QoL [23].

Our results showed that the QoL of the children in SEN group was significantly lower than their peers in various subscales for the senior age group. This finding may be due to peer pressure, which increases along with age [26]. The children from the senior age group were in the adolescent stage. Hormonal developments in the adolescent stage may create imbalances in physiological processes that have impacts on their subjective physical well-being [27]. Young adolescents also begin seeking their own identities and undergo the process of individualization, during which they experience uncertainty about the future. This unsettled condition imposes a health-related burden on adolescents. As mentioned, the children with SEN in general exhibited significantly lower scores in physical and social functioning than those with TD. This discrepancy may become aggravated with age, thus resulting in a higher sense of insecurity for the senior SEN age group than the junior SEN age group.

Furthermore, our results showed that the number of subscales for which those with SEN exhibited significantly lower QoL scores than those with TD was higher for the boys than for the girls. This result is consistent with another study in which boys in the SEN group exhibited more negative symptoms than girls with SEN [28]. In another study, boys with SEN reported a lower overall self-perception than their peers, and there were gender differences noted as well. Whereas boys tend to be more physically active and have stronger physical self-perception than girls, the physical limitations may impact boys more negatively than girls with SEN [29]. According to the literature, externalizing behaviors such as inattention and impulsivity may affect the behavior and learning of boys with SEN more significantly than girls, hence resulting in poorer academic performance and lower self-esteem [28]. This is consistent with our study that boys in the SEN group perceived a significantly lower school and psychosocial functioning than the girls.

### 4.3. Comparison of Parent and Child Agreement

Our study revealed significant differences in the perceptions of school functioning between the children and their parents in the SEN group. The mean score of school functioning reported by the children with SEN was higher than that reported by their parents. This finding is consistent with the previous studies that found discrepancies between children's and their parents' perceptions of the nonphysical QoL of the children with disabilities [15, 30]. One study proposed that parents' overexaggeration of their children's weaknesses was another reason for this underestimation [15]. Parents may compare their children with children with typical development and may be concerned more about their children's futures, regarding their peer relationships and academic achievement, causing them to underestimate their children's psychosocial QoL.

Studies have explained that children with ADHD might be overoptimistic in areas in which they have low performance, causing an overestimation of their functioning. This overoptimism is described as the positive illusion bias [31]. Children with ADHD tended to overestimate their performance to obtain a favorable internal representation of competencies as a self-protective mechanism [32]. This overoptimistic view may have led them to report higher scores on their psychosocial behaviors in our study, resulting in mean scores on school functioning that were higher than those reported by their parents. Discrepancies in parents' and children's perceptions of school functioning for children with SpLD can be explained by parents' negative perception of their children's academic performance, thus causing them to underestimate their children's school functioning [30]. Hong Kong parents greatly value academic excellence and have higher expectations of their children to perform well and achieve academic success than the children themselves [23]. This parental concern about achieving academic excellence may result in lower scores on the perception of QoL in terms of school functioning among parents of children with SpLD than among the children themselves.

### 4.4. Implications for Occupational Therapy

The findings of the study support the use of the Chinese version of PedsQL™ 4.0 Generic Module, including the child self-report and parent proxy report forms, to measure and compare the HRQOL of children and adolescents in Hong Kong. The study contributes to the initial establishment of local norms for the Chinese PedsQL, which can be used as outcome measures by healthcare professionals, including OT clinicians. Using the results obtained from the self-reports of clients, OT clinicians can focus on the domains with low scores to increase their engagement and their self-efficacy in meaningful occupations. Occupational therapists may use PedsQL to identify specific problem areas and formulate tailor-made interventions which can alleviate the difficulties faced by clients. Occupational therapists can also assist clients in identifying specific occupations that they value and develop interventions that are meaningful to them, thereby enhancing the clients' QoL [33]. By using PedsQL, a better understanding of clients' challenges in participation can be facilitated, which enhances the delivery of intervention.

### 4.5. Limitations

A small sample size with 48 children with TD and 21 children with SEN included in the study may affect the statistical power of the study. Convenience sampling was used to select the schools from which the participants were recruited, which may reduce the generalizability of our results to the overall population [23]. Further, face-to-face surveys were conducted for the SEN group to address any problems encountered by the participants immediately while filling the forms, whereas paper questionnaires and online surveys were used for the typically developing group. Different data collection formats may affect the validity of the results.

Future work can expand the sample size to increase the statistical power of the results. Random sampling methods should be adopted for higher generalization power. In addition, other environmental factors can be considered, such as family context, financial status, and the extent to which a family supports the measurement of their children's QoL [15]. While measuring QoL, the parents' knowledge of the disorders that their children are diagnosed with should be studied to increase the accuracy of the parents' perception of their children's QoL. Finally, to enhance the internal consistency reliability of the items, the overlapping of the subitems with disorder symptoms should be avoided when rating the QoL of children with SEN [20].

## 5. Conclusion

This research studied the HRQOL of local children in Hong Kong using the outcome measures of the Chinese version of PedsQL™ 4.0 Generic Module. The children with SEN reported a lower QoL in the physical and psychosocial domains and a lower overall score than the children with TD. The parents of both the typical development and the children with SEN in general perceived their children's QoL in a manner consistent with how the children themselves perceived it. Our findings provide preliminary indications that the Chinese version of PedsQL™ 4.0 is reliable and valid for the Hong Kong population and can be adopted for pediatric clinical and research purposes in the population.

## Figures and Tables

**Table 1:** Sociodemographic characteristics of the child participants.

Characteristics		Children with SEN (*N* = 21)	Children with TD (*N* = 48)
Mean age (SD)		8.80 (1.45)	10.08 (1.61)
Age group (%)	Junior (aged 7–8 years)	13 (61.9%)	14 (29.2%)
	Senior (aged 9–12 years)	8 (38.1%)	34 (70.8%)

Gender (%)	Male	12 (42.9%)	20 (58.3%)
	Female	9 (57.1%)	28 (41.7%)

Geographical regions (%)	Hong Kong Island	0	0
	Kowloon	16 (76.2%)	9 (18.8%)
	New territories	5 (23.8%)	39 (81.3%)

Diagnostic status (%)	Suspected/pending diagnosis	8 (38.1%)	
	Confirmed diagnosis	13 (61.9%)	

Diagnosis (%)	ADHD	7 (33.3%)	
	SpLD	5 (23.8%)	
	Developmental delay	1 (4.8%)	
	Others	3 (14.3%)	
	Comorbidity	5 (23.8%)	

Note. ADHD: attention deficit/hyperactivity disorder; SpLD: specific learning difficulty; SEN: special educational need; TD: typical development.

**Table 2:** Sociodemographic characteristics of parent participants.

		Parents of children with SEN (*N* = 21)	Parents of children with TD (*N* = 48)
Mean age (SD)	Father	40.33 (19.1)	42.90 (10.2)
	Mother	41.14 (7.13)	38.85 (7.84)

Paternal educational level (%)	Primary	2 (9.52%)	4 (8.33%)
	Junior secondary	4 (19.0%)	18 (37.5%)
	Senior secondary	6 (28.6%)	16 (33.3%)
	High diploma	4 (19.0%)	1 (2.08%)
	University	3 (14.3%)	9 (18.8%)
	Missing data	2 (9.52%)	0

Maternal educational level (%)	Primary	3 (14.3%)	2 (4.17%)
	Junior secondary	6 (28.6%)	17 (35.4%)
	Senior secondary	7 (33.3%)	17 (35.4%)
	High diploma	1 (4.76%)	8 (16.7%)
	University	4 (19.0%)	4 (8.33%)

Note. SEN: special educational needs; TD: typical development.

**Table 3:** Internal consistency reliability of the scale and its subscales between TD and SEN children and parent groups.

		*N*	Cronbach's alpha (*α*)
Physical health	Children with SEN	21	0.739
	Parents of children with SEN		0.915
	Children with TD	48	0.724
	Parents of children with TD		0.853

Emotional functioning	Children with SEN	21	0.611
	Parents of children with SEN		0.656
	Children with TD	48	0.823
	Parents of children with TD		0.847

Social functioning	Children with SEN	21	0.721
	Parents of children with SEN		0.826
	Children with TD	48	0.826
	Parents of children with TD		0.897

School functioning	Children with SEN	21	^∗^0.480
	Parents of children with SEN		^∗^0.566
	Children with TD	48	0.775
	Parents of children with TD		0.835

Psychosocial health^∗∗^	Children with SEN	21	0.812
	Parents of children with SEN		0.854
	Children with TD	48	0.895
	Parents of children with TD		0.925

Overall score	Children with SEN	21	0.878
	Parents of children with SEN		0.867
	Children with TD	48	0.904
	Parents of children with TD		0.937

*Note.* ^∗^ *α* ≤ 0.5: unacceptable internal consistency; ^∗∗^the psychosocial health subscale is the mean of the emotional, social, and school subscales. SEN: special educational needs; TD: typical development.

**Table 4:** Comparison of PedsQL between children with SEN and TD.

		*n*	Mean (SD)	*p*
Physical health	SEN group	21	74.26 (17.48)	^∗^0.000
	TD group	48	90.36 (10)	

Emotional functioning	SEN group	21	69.52 (18.97)	0.183
	TD group	48	76.04 (18.65)	

Social functioning	SEN group	21	75.57 (21.77)	0.012
	TD group	48	89.17 (13.77)	

School functioning	SEN group	21	68.57 (17.04)	0.012
	TD group	48	78.85 (16.38)	

Psychosocial health^∗∗^	SEN group	21	71.22 (16.08)	0.015
	TD group	48	81.35 (13.87)	

Overall score	SEN group	21	72.27 (15.72)	^∗^0.002
	TD group	48	84.49 (11.50)	

Note. ^∗^*p* < 0.05; ^∗∗^psychosocial health subscale: the mean scores of the emotional, social, and school subscales. SEN: special educational needs; TD: typical development.

**Table 5:** Age comparison of PedsQL between children with SEN and TD.

Variables	Mean (SD) scores on subscales					
	Physical health	Emotional functioning	Social functioning	School functioning	Psychosocial health^∗∗∗^	Overall score
Junior age group (ages 7 to 8)						
SEN group (*n* = 13)	75 (16.54)	70 (17.32)	81.54 (21.64)	68.85 (16.73)	73.46 (15.45)	74.00 (14.91)
TD group (*n* = 14)	91.52 (11.91)	77.86 (14.10)	83.93 (15.46)	75.71 (17.53)	79.17 (13.69)	83.46 (12.43)
*p*	^∗∗^0.008	0.461	1.000	0.129	0.343	0.064

Senior age group (ages 9 to12)						
SEN group (*n* = 8)	73.05 (20.04)	68.75 (22.64)	65.88 (19.43)	68.13 (18.70)	67.58 (17.47)	69.48 (17.63)
TD group (*n* = 34)	89.89 (9.27)	75.29 (20.37)	91.32 (12.63)	80.15 (15.98)	82.25 (14.04)	84.91 (11.27)
*p*	^∗^0.034	0.326	^∗∗^0.001	0.076	^∗^0.034	^∗^0.023

Note. ^∗^*p* < 0.05; ^∗∗^*p* < 0.01; ^∗∗∗^psychosocial health subscale: the mean scores of the emotional, social, and school subscales. SEN: special educational needs; TD: typical development.

**Table 6:** Gender comparison of PedsQL between children with SEN and TD.

Variables	Mean (SD) scores on subscales					
	Physical health	Emotional functioning	Social functioning	School functioning	Psychosocial health^∗∗∗^	Overall score
Girls with SEN and TD						
SEN group (*n* = 9)	75.35 (19.10)	67.22 (18.05)	70.78 (21.14)	76.11 (18.50)	71.37 (16.32)	72.75 (16.41)
TD group (*n* = 28)	89.51 (9.36)	72.14 (18.28)	88.75 (13.45)	76.25 (17.57)	79.05 (13.43)	82.69 (10.93)
*p*	0.060	0.393	^∗^0.025	0.844	0.184	0.141

Boys with SEN and TD						
SEN group (*n* = 12)	73.44 (16.99)	71.25 (20.24)	79.17 (22.45)	62.92 (14.05)	71.11 (16.63)	71.92 (15.91)
TD group (*n* = 20)	91.56 (10.97)	81.5 (18.22)	89.75 (14.55)	82.5 (14.19)	84.58 (14.16)	87.01 (12.09)
*p*	^∗∗^0.002	0.170	0.103	^∗∗^0.001	^∗^0.020	^∗∗^0.006

Note. ^∗^*p* < 0.05; ^∗∗^*p* < 0.01; ^∗∗∗^psychosocial health subscale: the mean scores of the emotional, social, and school subscales. SEN: special educational needs; TD: typical development.

**Table 7:** Parent–child agreement on PedsQL.

		*N*	Mean score (SD)	*p*
Physical functioning	Children with SEN	21	74.26 (17.48)	0.478
	Parents of children with SEN		77.68 (17.15)	
	Children with TD	48	90.36 (10)	0.173
	Parents of children with TD		86.33 (13.28)	

Emotional functioning	Children with SEN	21	69.52 (18.97)	0.210
	Parents of children with SEN		62.65 (15.88)	
	Children with TD	48	76.04 (18.65)	0.565
	Parents of children with TD		78.33 (16.45)	

Social functioning	Children with SEN	21	75.57 (21.77)	0.117
	Parents of children with SEN		65.24 (19.52)	
	Children with TD	48	89.17 (13.77)	0.720
	Parents of children with TD		88.33 (14.74)	

School functioning	Children with SEN	21	68.57 (17.04)	0.058
	Parents of children with SEN		59.29 (14.17)	
	Children with TD	48	78.85 (16.38)	0.924
	Parents of children with TD		78.96 (17.35)	

Psychosocial health^∗^	Children with SEN	21	71.22 (16.08)	0.066
	Parents of children with SEN		62.39 (14.01)	
	Children with TD	48	81.35 (13.87)	0.820
	Parents of children with TD		81.88 (14.21)	

Overall functioning	Children with SEN	21	72.27 (15.72)	0.378
	Parents of children with SEN		67.71 (11.88)	
	Children with TD	48	84.49 (11.50)	0.837
	Parents of children with TD		83.42 (12.88)	

Note. ^∗^The psychosocial subscale is the mean of the emotional, social, and school subscales. SEN: special educational needs; TD: typical development.

## Data Availability

The data used to support the findings of this study are available from the corresponding author upon request.
